This article has been retracted.

# Silver Trimolybdate (Ag_2_Mo_3_O_10_.2H_2_O) Nanorods: Synthesis, Characterization, and Photo-Induced Antibacterial Activity under Visible-Light Irradiation

**DOI:** 10.1155/2022/2260083

**Published:** 2022-07-09

**Authors:** Maria Karollyna do Nascimento Silva Leandro, João Victor Barbosa Moura, Ana Carolina Justino de Araújo, Priscilla Ramos Freitas, Cicera Laura Roque Paulo, Amanda Karine de Sousa, Janaina Esmeraldo Rocha, Lívia Maria Garcia Leandro, Rakel Olinda Macedo da Silva, Clenilton Costa dos Santos, Jaime Ribeiro-Filho, Cleânio da Luz Lima, Abolghasem Siyadatpanah, Zahra Seifi, Bonglee Kim, Henrique Douglas Melo Coutinho

**Affiliations:** ^1^Laboratório de Microbiologia e Biologia Molecular-LMBM, Universidade Regional do Cariri—URCA, Crato, Ceará, Brazil; ^2^Centro Universitário Dr. Leão Sampaio-Unileão Juazeiro do Norte, Juazeiro do Norte, Ceará, Brazil; ^3^Departamento de Física, Centro de Ciências Exatas e Tecnologias, Universidade Federal do Maranhão—UFMA, São Luís, Maranhão, Brazil; ^4^Instituto Gonçalo Moniz, Fundação Oswaldo Cruz, IGM-FIOCRUZ/BA, Salvador, Bahia, Brazil; ^5^Departamento de Física, Centro de Ciências da Natureza, Universidade Federal do Piauí—UFPI, Teresina, Piauí, Brazil; ^6^Ferdows School of Paramedical and Health, Birjand University of Medical Sciences, Birjand, Iran; ^7^Laboratory Sciences Research Center, Golestan University of Medical Sciences, Gorgan 49189-36316, Iran; ^8^Department of Pathology, College of Korean Medicine, Kyung Hee University, Seoul 02447, Republic of Korea; ^9^Korean Medicine-Based Drug Repositioning Cancer Research Center, College of Korean Medicine, Kyung Hee University, Seoul 02447, Republic of Korea

## Abstract

The present study reports the synthesis, characterization, and antibacterial properties of silver trimolybdate (Ag_2_Mo_3_O_10_.2H_2_O) nanorods. The synthesis was performed using a conventional hydrothermal method. The sample was characterised by scanning electron microscopy (SEM), X-ray diffraction (XRD), Fourier transform infrared (FTIR) spectroscopy, UV–Vis–NIR diffuse reflectance, thermogravimetric analysis (TGA), and differential scanning calorimeter (DSC). The direct antibacterial activity was evaluated using the microdilution method to determine the minimum inhibitory concentration (MIC). To assess the ability of Ag_2_Mo_3_O_10_.2H_2_O nanorods to modulate antibacterial resistance, the MIC of aminoglycosides was established in the presence of a subinhibitory concentration of this substance alone and associated with LED light exposure. The characterization of the sample indicated that the synthesis of silver trimolybdate generated nanometric crystals with rod-like morphology, without secondary phases. The treatment with Ag_2_Mo_3_O_10_.2H_2_O nanorods alone or combined with visible LED lights exhibited clinically relevant antibacterial activity against both Gram-negative and Gram-positive bacteria. This nanostructure presented a variable antibiotic-modulating action, which was not improved by visible LED light exposure. Nevertheless, LED lights showed promising antibiotic-enhancing activities in the absence of Ag_2_Mo_3_O_10_.2H_2_O nanorods. In conclusion, silver trimolybdate dihydrate nanorods have antibacterial properties that can be photocatalysed by visible-light exposure. While showing the potential use to combat antibacterial resistance, the simultaneous combination of silver trimolybdate, visible LED lights, and antibacterial drugs should be carefully analysed to avoid antagonist effects that could impair the effectiveness of antibiotic therapy.

## 1. Introduction

The molybdates, a group of inorganic substances belonging to the family of transition-metal oxides, are formed by combining the [MoO_4_]^2−^ ion with different cations. Studies have demonstrated that these substances present unique physical properties such as ferroelasticity and ferroelectricity, making them suitable for synthesising substances with various sizes, morphologies, and applications [1].

Accordingly, metallic molybdates with variable chemical and structural characteristics have been synthesised and assessed for biological activities in different fields of investigation [2, 3]. In this context, silver molybdates such as Ag_2_MoO_4_, Ag_2_Mo_2_O_7_, and Ag_2_Mo_3_O_10_ can be obtained as crystalline structures by combining molybdenum anions with silver cations. Importantly, consistent evidence has demonstrated that these compounds present remarkable antibacterial properties, which indicate that they have the potential to be used in targeted drug development to overcome bacterial resistance [4–6].

These nanoscale material systems have been highlighted in several scientific studies as a possible alternative to combat resistant microorganisms, since they have a very small size, but a large surface area, and are able to improve the delivery of drugs in specific tissues. These characteristics lead to increased efficacy and decreased adverse effects of antimicrobials by controlling the dosage and time of action [7].

The discovery of novel compounds with bactericidal and bacteriostatic properties has gained increasing attention as the rise of bacterial resistance to conventional antibiotics has impaired the treatment of both community and hospital infections [8]. Also, researchers have developed new strategies to potentiate the activity of antibiotics against resistant bacteria, including the association of conventional drugs with new chemical entities and light-emitting diode (LED) lights [9, 10]. In this context, previous research has demonstrated that silver molybdates present a photocatalytic activity [11]. Accordingly, it was reported that *β*-Ag_2_MoO_4_ exhibited potent photocatalytic activity concerning the degradation of ciprofloxacin, which might be related to the absorption of visible UV light [12].

The WHO (World Health Organization) encourages the governments of various countries to support studies for the development of effective and low-cost antibiotics, since the pharmaceutical industry has encountered scientific and economic difficulties during the development of these drugs [13]. Therefore, considering the evidence that silver molybdates could modulate bacterial resistance [14–16], this study aims to investigate the antibacterial, antibiotic-enhancing, and photocatalytic activities of silver trimolybdate dihydrate (Ag_2_Mo_3_O_10_.2H_2_O) nanorods against resistant strains of *Staphylococcus aureus* and *Escherichia coli* in association with visible LED lights.

## 2. Materials and Methods

### 2.1. Synthesis and Characterization of Ag_2_Mo_3_O_10_.2H_2_O Nanorods

Silver trimolybdate dihydrate (Ag_2_Mo_3_O_10_.2H_2_O) nanorods were synthesised using a simple hydrothermal method, as described previously [17]. In brief, 0.1062 g of silver nitrate (AgNO_3_) and 0.2194 g of ammonium heptamolybdate tetrahydrate ((NH_4_)_6_Mo_7_O_24_.4H_2_O) were dissolved in 20 mL of deionised water. These solutions were then mixed, and the pH was adjusted to 2 with HNO_3_. The resulting solution was transferred to a 50 mL Teflon-lined stainless autoclave and maintained at 140°C for 6 h. The yellowish precipitates were repeatedly washed with deionised water using a centrifuge at 3600 rpm for 15 minutes and dried in an air oven at 70°C for 12 h.

The morphological aspects of the samples were analysed by scanning electron microscopy (SEM). The SEM images were obtained using a Tescan Vega 3 SBU scanning electron microscope. The structural characterization was performed by X-ray diffraction (XRD) using a Mini-Flex Rigaku diffractometer equipped with Cu K*α* (*λ* = 1.5418 Å) radiation in the 2*θ* range of 10°–80°, with a step size of 0.02° and a count time of 2 s/step. Fourier transform infrared (FTIR) spectra were taken from 4000 to 450 cm^−1^ using KBr pellets as a reference using a Perkin Elmer Spectrum Two spectrophotometer in transmittance mode. Thermogravimetric analysis (TGA) and differential scanning calorimetry (DSC) data were obtained using a simultaneous thermal analysis equipment, STA 449 F3 Jupiter by Netzsch. A heating rate of 10°C·min^−1^ was selected to measure the sample under a stream of nitrogen (100 mL·min^−1^), between 25 and 600°C, using Al_2_O_3_ open capsules. The UV–Vis–NIR diffuse reflectance measurements were performed using a Shimadzu UV-3600 spectrophotometer equipped with an integrating sphere accessory (model ISR-3100). Diffuse reflectance analysis was used to estimate the band gap of the compound.

### 2.2. Antibacterial Activity Analysis

The standard (*E. coli* ATCC 25922 and *S. aureus* ATCC 25923) and multidrug-resistant (*S. aureus* 10 and *E. coli* 06) bacterial strains used in this study were provided by the Laboratory of Microbiology and Molecular Biology (LMBM) from the Regional University of Cariri (URCA). The antibiotics amikacin and gentamicin, as well as all reagents used in the tests, were purchased from Sigma Chemical Co. (St. Louis, USA). All drugs were diluted in distilled water to an initial concentration of 1024 *μ*g/mL.

The MIC of each drug was determined using the broth microdilution method. All strains were cultured in a heart infusion agar (HIA) solid medium for 24 h at 37°C. Samples were transferred from the solid medium to test tubes containing sterile saline, and turbidity was assessed using a value of 0.5 on the McFarland scale. Each inoculum was prepared with 10% BHI (brain heart infusion) to obtain a dilution of 1 : 9. Next, 100 *μ*L of inoculum in the medium was transferred to wells on a 96-well plate with 100 *μ*L of the drugs at concentrations ranging from 512 to 8 *μ*g/mL, followed by incubation at 37°C for 24 h. Wells containing only the inoculum in BHI were used as a growth control [18–20]. After incubation, 20 *μ*L of 0.01% sodium resazurin solution was added to each well, followed by incubation for 1 h at room temperature. A change in the color of the solution from blue to red indicated bacterial growth. The MIC was defined as the lowest concentration capable of inhibiting bacterial growth [21]. All experiments were carried out in triplicate.

### 2.3. Analysis of Antibiotic Resistance Modulation by Ag_2_Mo_3_O_10_.2H_2_O Nanorods

The antibiotic-enhancing activity was evaluated using the methodology described by Coutinho and collaborators [19]. To this end, the bacterial inocula were prepared in BHI as described above, and Ag_2_Mo_3_O_10_.2H_2_O nanorods were added at a subinhibitory concentration (equivalent to its MIC: 8 *μ*g/mL). All wells on a 96-well plate were filled with 100 *μ*L of this solution, followed by adding 100 *μ*L of each antibiotic at concentrations ranging from 512 to 0.5 *μ*g/mL. The MIC of each drug was determined, and the occurrence of synergism was interpreted as an enhanced antibiotic activity. Experimental controls and readings were performed as previously described.

### 2.4. Evaluation of Antibiotic-Modulating Activity in Association with LED Light Exposure

A light emitting diodes (LEDs) device (NEW Estética®) was used in the experimental protocols. This device allows illuminating the samples with red (620 nm), yellow (590 nm), and blue (415 nm) colored light and also a combination of these colors; the wavelength is predetermined by the apparatus.

To evaluate the effect of LED light exposure on bacterial growth on antibacterial activity modulation, cultures and treatments were carried out as previously described. The plates were exposed to either blue, red, or yellow light for 20 min and then incubated at 37°C for 24 h. Plates without LED light exposure were used as experimental controls. The readings were performed as described before.

### 2.5. Statistical Analysis

Data are expressed as mean ± standard deviation, and differences were evaluated through analysis of variance (ANOVA) followed by Bonferroni's post hoc test using the GraphPad Prism 6.0 software. The differences with *p* < 0.05 were considered significant.

## 3. Results and Discussion

Morphology of the as-prepared Ag_2_Mo_3_O_10_.2H_2_O nanorods was evaluated by the SEM technique. Figures 1(a) and 1(b) show the SEM images of the sample in low and high magnifications, respectively. Figures 1(a) and 1(b) show that the material formed has unique straight rod-like structures without links between rods. In addition, the as-prepared material presented high morphology homogeneity. Amorphous materials or aggregates were not detected, confirming that the synthesis procedure using the hydrothermal method resulted in a sample of excellent purity and quality. The diameter size distribution histogram (Figure 1(c)) of the nanorods shows that the average diameter size obtained is 136 nm (range of 54–350 nm).

The XRD pattern of the samples obtained in the present study is shown in Figure 2. The crystalline nature of the Ag_2_Mo_3_O_10_.2H_2_O nanorods was confirmed by XRD analysis. The respective positions of diffraction peaks in the XRD pattern found are in good agreement with the results reported by the Inorganic Crystal Structure Database (ICSD) N° 162219, indicating the formation of Ag_2_Mo_3_O_10_.2H_2_O crystals with orthorhombic structure and space group *D*_2h_^16^ (*Pnma*), without secondary phases. The sharp and well-defined diffraction peaks indicated a high degree of structural order and crystallinity at the long-range, proving the effectiveness of the synthesis method employed in this work.

The FTIR spectrum of Ag_2_Mo_3_O_10_.2H_2_O nanorods at atmospheric conditions in the spectral range between 4500 and 450 cm^−1^ is shown in Figure 3. The vibrational bands between 500 and 1000 cm^−1^ were assigned to the stretching modes of Ag_2_Mo_3_O_10_.2H_2_O. The peak around 1625 cm^−1^ and the broadband between 3000 and 3500 cm−1 were attributed, respectively, to the bending and stretching vibrations of the H_2_O molecules, both connected to Ag_2_Mo_3_O_10_.2H_2_O (crystallised water) and adsorbed on the surface of the nanorods. The relative positions of all infrared modes of silver trimolybdate dihydrate nanorods are consistent with the literature data, confirming the results of the XRD analysis [17].

Figure 4 shows the mass changes and heat flow rate of the thermal modifications of Ag_2_Mo_3_O_10_.2H_2_O nanorods determined by thermogravimetric analysis (TGA) and differential scanning calorimetry (DSC) techniques. Following the characterization of the Ag_2_Mo_3_O_10_.2H_2_O nanorods, the DSC analysis shows four events (Figure 4). The first endothermic event occurs at temperatures below 100°C and corresponds to the loss of adsorbed water on the surface of the nanorods. The second endothermic event occurs at approximately 250°C and corresponds to the loss of crystallised water in the sample. A third event is observed at around 335°C and indicates a structural phase transition of Ag_2_Mo_3_O_10_.2H_2_O. The last endothermic event occurs at about 530°C, corresponding to the decomposition of the sample. Two distinct mass loss steps were detected in the TGA curve. The first thermal event, around 65–120°C, with a mass loss of 0.5%, is attributed to the loss of adsorbed water on the surface of the nanorods. The second thermal event, which occurs between 230 and 70°C, with a mass loss of 0.5%, corresponds to the loss of crystallised water in the Ag_2_Mo_3_O_10_.2H_2_O nanorods. The DSC and TGA results are in excellent agreement and indicate that the sample has a wide range of thermal stability and, as such, can be used in thermal processes that involve the production of antibacterial composites.

The energy gap (*E*_gap_) of Ag_2_Mo_3_O_10_.2H_2_O nanorods can be estimated by extrapolating the linear part of Kubelka–Munk function, which is the ratio between the absorption and scattering factor from the optical diffuse reflectance spectrum [22]. Based on UV–visible diffuse reflectance measurements, a plot of (F(R)h*ν*)^1/2^ versus photon energy (h*ν*) is shown in Figure 5, where it can be seen that Ag_2_Mo_3_O_10_.2H_2_O nanorods present a band gap energy (*E*_gap_) of about 2.80 eV. The *E*_gap_ obtained is similar to that reported in the literature [17] and is located in the visible spectrum. The ability to absorb visible light makes this material promising for research with photocatalytic activity.

The antibacterial activity analysis results, given in Table 1, demonstrated that silver trimolybdate alone exerted a moderate action against standard and multidrug-resistant strains of *S. aureus* and *E. coli*, with no significant variation among these strains. Exposure to different LED lights resulted in variable changes in the MIC of this compound. While exposure to yellow light resulted in significantly increased antibacterial activity of silver trimolybdate against the standard *S. aureus* strain, it does not affect the activity of this substance against the corresponding resistant strain. In addition, all other combinations of LED lights and Ag_2_Mo_3_O_10_.2H_2_O nanorods showed antagonistic effects, indicating decreased antibacterial activity. Therefore, only yellow light was found to present clinically valuable results concerning the modulation of silver trimolybdate antibacterial activity. It is worth mentioning that this is the first study reporting the antibacterial activity of Ag_2_Mo_3_O_10_.2H_2_O nanostructures.

The antibacterial activity demonstrated by silver trimolybdate dihydrate is corroborated by previous studies demonstrating a significant action of *β*-Ag_2_MoO_4_ crystals against *E. coli* [16]. In addition, different compounds obtained as silver molybdate crystals have demonstrated significant activities against both Gram-positive and Gram-negative bacteria [15], as well as against fungal strains [23]. However, the mechanisms of action underlying the antibacterial effects of crystals containing silver atoms remain to be fully characterised. Nevertheless, it has been suggested that the chemical properties of these compounds favor their interaction with the negatively charged peptidoglycan wall, which could result in increased cell permeability, followed by cell disruption and bacterial death [24]. In addition, since bacterial cells present elevated concentrations of sulfur and phosphorus, the binding of these compounds to organelles containing these elements could lead to impaired cellular respiration and DNA denaturation, resulting in inhibition of crucial processes for bacterial growth [25]. Accordingly, Ali and collaborators [26] reported that the antibacterial effect of Ag-doped TiO_2_ nanoparticles was associated with the production of hydroxyl radicals, which mediated the formation of pores in the bacterial cell membrane.

These results obtained are promising considering that the pharmaceutical area is one of the most involved with the study and development of nanoparticles, since they can present different biological actions in the human body, either by direct contact or by incorporation with other products, being the main routes of entry into the body: the skin (topical use), the lung (inhalation), and the gastrointestinal tract (ingestion) [27].

Concerning the events observed in the present study, the generation of potent oxidative agents, including the superoxide ion (O_2_'), OOH^*∗*^ radicals, and hydrogen ions (H•), could occur as a consequence of electron-hole transfer in the bulk-surface interface [16]. Therefore, oxidation of macromolecules such as lipids, proteins, and nucleic acids could lead to significant cytotoxicity [28]. Since Ag_2_Mo_3_O_10_.2H_2_O nanorods present a bandgap in the visible spectrum region (Figure 5), they can absorb visible light, which in turn induces the formation of free radicals generated by the transfer of electron-hole pairs on the surface of the nanocrystals. Therefore, considering evidence that this substance presents photocatalytic properties [17], we analysed its antibiotic-enhancing properties associated with exposure to visible LED light.

An analysis of the photocatalytic effect of LED lights in association with Ag_2_Mo_3_O_10_.2H_2_O nanorods demonstrated that exposure to blue and red LED lights resulted in no clinically useful modulation of the antibacterial activity. In addition, some combinations resulted in antagonistic effects that could be harmful in antimicrobial therapy. Nevertheless, exposure to yellow light resulted in significantly increased antibacterial activity of silver trimolybdate nanorods against the standard *S. aureus* strain. This finding corroborated previous research showing that exposure to visible light increased the activity of graphitic carbon nitride incorporated into silver nanoparticles against *S. aureus* [29].

Following the antibacterial activity analysis, this study evaluated the ability of Ag_2_Mo_3_O_10_.2H_2_O nanorods to reverse bacterial resistance against amikacin and gentamicin. As shown in Figure 6, the compound significantly decreased the MIC of both antibiotics against the Gram-negative strain. However, in the tests with *S. aureus*, the association with a subinhibitory concentration of silver trimolybdate nanorods caused no change in the MIC of amikacin, besides increasing the MIC of gentamicin. Therefore, these findings suggest that Ag_2_Mo_3_O_10_.2H_2_O nanorods reverted, at least partially, the degree of observed resistance to aminoglycosides in *E. coli*, which was not found in *S. aureus*.

The synergism observed in the association between the silver trimolybdate nanorods and the aminoglycoside antibiotics represent a promising finding in targeted research for antibacterial drug development. Evidence has pointed to a massive increase in antibacterial resistance in *E. coli* strains [19]. In this context, chemical compounds containing silver have attracted considerable attention in antimicrobial therapy, as they exert a direct antibacterial activity associated with minimal induction of antibacterial resistance [30]. According to Smekalova and collaborators [31], the interaction between silver atoms and the peptidoglycan layer is favored in Gram-negative strains due to its thinner and less rigid structure than in Gram-negative bacteria. Thus, according to this hypothesis, the interaction with the peptidoglycan would facilitate the penetration of the aminoglycosides, justifying their enhanced antibacterial activity against *E. coli*.

As we demonstrated that LED light exposure differentially modulated the antibacterial activity of silver trimolybdate nanorods, which in turn presented antibiotic-modulating properties in association with aminoglycosides, this study investigated the antibiotic-modulating effects of LED light exposure associated or not with Ag_2_Mo_3_O_10_.2H_2_O nanorods (Figures 7(a)–7(c)). Exposure to the blue LED light (A) potentiated the effects of gentamicin against both strains, which was not found for amikacin. However, in the presence of a subinhibitory concentration of Ag_2_Mo_3_O_10_.2H_2_O nanorods, no improvement in antibiotic activity was observed, and most associations resulted in antagonistic effects. On the other hand, the yellow LED light (B) potentiated the action of both antibiotics against *E. coli*, as well as potentiated the action of gentamicin in front of *S. aureus*. However, in the presence of Ag_2_Mo_3_O_10_.2H_2_O, both drugs presented reduced antibacterial activities against resistant strains of *E. coli* and *S. aureus*. Finally, exposure to the red LED light (C) increased the activity of amikacin and gentamicin against *E. coli* and *S. aureus*, respectively. However, when simultaneously combined with Ag_2_Mo_3_O_10_.2H_2_O nanorods and irradiated with the red light, both drugs had their MIC against *S. aureus* increased.

Studies have indicated that the antibacterial and antibiotic-modulating activities of LED lights are due to photodynamic inactivation of microorganisms that results from the generation of reactive oxygen species as a consequence of the interaction between the emitted light and the photosensitising agent [32]. Therefore, the association of aminoglycosides with LED lights may represent a promising strategy for treating skin infections caused by resistant bacteria. Notably, the development of target research aimed at optimising the applications of microorganism photoinactivation can significantly contribute to advances in combined therapy for bacterial diseases [33].

The present study results show that different wavelengths in the visible spectrum can potentiate the action of aminoglycosides against both Gram-positive and Gram-negative strains. However, the simultaneous association with Ag_2_Mo_3_O_10_.2H_2_O nanorods seems to interfere with the biochemical mechanisms involved in this phenomenon, impairing antibacterial action. In addition, it has been demonstrated that, due to the photocatalyst effect, Ag_2_Mo_3_O_10_.2H_2_O nanorods can induce the degradation of organic compounds such as strains, as well as the antibiotics used. It is well known in the literature that the Ag_2_Mo_3_O_10_.2H_2_O nanostructured is an efficient visible-light-driven plasmonic photocatalyst for the degradation of glyphosate and rhodamine B dye, which shows high efficiency in the degradation of organic compounds [17, 34].

Liu et al. [35] synthesised Ag_2_Mo_3_O_10_ 1.8H_2_O with rod-like structures by chemical precipitation, and after this obtaining, AgI/Ag_2_Mo_3_O_10_·1.8H_2_O was subsequently formed. In tests to evaluate the photocatalytic activity of this material, efficient results in dye degradation were also obtained.

Thus, significant degradation of aminoglycosides could justify the frequent antagonistic effects resulting from the simultaneous association with Ag_2_Mo_3_O_10_.2H_2_O nanorods and visible LED lights.

Other studies have already reported these photocatalytic effects of antibiotics, such as the degradation of norfloxacin hydrochloride [36], gentamicin [37], and amikacin [38], so it becomes increasingly important, studies of synthesis and application of nanostructured materials for environmental recovery, since the inefficiency of effluent treatment methods or even the absence of these in municipalities, associated with the exacerbated consumption of antibiotics, contribute to the ubiquity of these drugs in various environments, especially aquatic, increasing the proliferation of multidrug-resistant bacteria and toxicity, which makes it essential, the development of new efficient tools to degrade these compounds [39].

## 4. Conclusion

The synthesis of Ag_2_Mo_3_O_10_.2H_2_O nanorods using a simple hydrothermal method generated nanometric crystals with rod-like morphology. The treatment with silver trimolybdate nanorods alone or combined with visible LED lights exhibited clinically relevant antibacterial activity against Gram-negative and Gram-positive bacteria. This nanomaterial presented a variable antibiotic-modulating action, which was not improved by LED light exposure. Nevertheless, visible LED lights showed promising antibiotic-enhancing activities in the absence of Ag_2_Mo_3_O_10_.2H_2_O nanorods.

In conclusion, silver trimolybdate nanorods have antibacterial properties that can be photocatalysed by visible-light exposure. While showing the potential be used to combat antibacterial resistance, the simultaneous combination of Ag_2_Mo_3_O_10_.2H_2_O nanorods, LED lights, and antibacterial drugs should be carefully analysed to avoid antagonist effects that could impair the effectiveness of antibiotic therapy.

## Figures and Tables

**Figure 1:** (a) Low and (b) high-magnification SEM images of Ag_2_Mo_3_O_10_.2H_2_O nanorods prepared by the hydrothermal method (magnifications: (a) 2 kx and (b) 10 kx). (c) The diameter size distribution of the nanorods.

**Figure 2:** X-ray diffraction pattern of the Ag_2_Mo_3_O_10_.2H_2_O nanorods obtained by the hydrothermal method.

**Figure 3:** FTIR spectrum of Ag_2_Mo_3_O_10_.2H_2_O nanorods.

**Figure 4:** Thermogravimetric (black) and differential scanning calorimetry (red) curves of Ag_2_Mo_3_O_10_.2H_2_O nanorods.

**Figure 5:** Diffuse reflectance ultraviolet–visible spectrum of Ag_2_Mo_3_O_10_.2H_2_O nanorods.

**Figure 6:** Minimum inhibitory concentration (MIC) of amikacin and gentamicin alone or in the presence of Ag_2_Mo_3_O_10_.2H_2_O, against multidrug-resistant strains of <i>S. aureus</i> and <i>E. coli</i>. ^*∗∗∗∗*^*P* < 0.0001 indicates significant differences between groups. Statistical significance was determined by one-way ANOVA and Bonferroni's post hoc test.

**Figure 7:** Minimum inhibitory concentration (MIC) of amikacin and gentamicin alone or in the presence of Ag_2_Mo_3_O_10_.2H_2_O and blue (a), yellow (b), or red (c) LED lights, against multidrug-resistant strains of *S. aureus* and *E. coli*. ^*∗∗∗∗*^*P* < 0.0001 indicates significant differences between groups. Statistical significance was determined by one-way ANOVA and Bonferroni's post hoc test.

**Table 1:** Minimum inhibitory concentration (MIC) of Ag_2_Mo_3_O_10_.2H_2_O.

Treatment	E.C ATCC 25922	S.A ATCC 25923	E.C 06	S.A 10
Ag_2_Mo_3_O_10_.2H_2_O	512	426.66	512	512
Ag_2_Mo_3_O_10_.2H_2_O + blue light	853,33	682.66	≥1024	≥1024
Ag_2_Mo_3_O_10_.2H_2_O + yellow light	≥1024	128	≥1024	512
Ag_2_Mo_3_O_10_.2H_2_O + red light	≥1024	512	≥1024	≥1024

S.A., *Staphylococcus aureus;* E.C., *Escherichia coli.* The MIC values are expressed in *μ*g/mL.

## Data Availability

The data used to support the findings of this study are available from the corresponding authors upon request.

## References

[1] Maczka M., Souza Filho A., Paraguassu W., Freire P., Mendes Filho J., Hanuza J. (2012). Pressure-induced structural phase transitions and amorphization in selected molybdates and tungstates. *Progress in Materials Science*.

[2] Yeo B. R., Pudge G. J., Bugler K. G. (2016). The surface of iron molybdate catalysts used for the selective oxidation of methanol. *Surface Science*.

[3] Moura J., Pinheiro G., Silveira J., Freire P., Viana B., Luz-Lima C. (2017). NaCe (MoO4) 2 microcrystals: hydrothermal synthesis, characterization and photocatalytic performance. *Journal of Physics and Chemistry of Solids*.

[4] Tang H., Fu Y., Chang S., Xie S., Tang G. (2017). Construction of Ag3PO4/Ag2MoO4 Z-scheme heterogeneous photocatalyst for the remediation of organic pollutants. *Chinese Journal of Catalysis*.

[5] Feng M., Zhang M., Song J.-M., Li X.-G., Yu S.-H. (2011). Ultralong silver trimolybdate nanowires: synthesis, phase transformation, stability, and their photocatalytic, optical, and electrical properties. *ACS Nano*.

[6] Tang H., Lu A., Li L., Zhou W., Xie Z., Zhang L. (2013). Highly antibacterial materials constructed from silver molybdate nanoparticles immobilized in chitin matrix. *Chemical Engineering Journal*.

[7] Lombardo D., Kiselev M. A., Caccamo M. T. (2019). Smart nanoparticles for drug delivery application: development of versatile nanocarrier platforms in biotechnology and nanomedicine. *Journal of Nanomaterials*.

[8] Silva A. C., Diodato J. S., Castro J. W. (2019). Effect of the essential oils from piper sp. and blue led lights in the enhancement of the antibiotic activity of drugs against mdr bacterial strains. *Journal of Photochemistry and Photobiology B: Biology*.

[9] Pereira N. L., Aquino P. E., Júnior J. G. (2017). Antibacterial activity and antibiotic modulating potential of the essential oil obtained from Eugenia jambolana in association with led lights. *Journal of Photochemistry and Photobiology B: Biology*.

[10] Ferreira Matias E. F. (2017). Avaliação da atividade antibacteriana e moduladora do óleo essencial de Cordia verbenacea DC. associado às luzes de LED. *Revista Interfaces: Saúde, Humanas e Tecnologia*.

[11] Kumar J. V., Karthik R., Chen S.-M., Muthuraj V., Karuppiah C. (2016). Fabrication of potato-like silver molybdate microstructures for photocatalytic degradation of chronic toxicity ciprofloxacin and highly selective electrochemical detection of H_2_O_2_. *Scientific Reports*.

[12] Bai Y.-Y., Lu Y., Liu J.-K. (2016). An efficient photocatalyst for degradation of various organic dyes: Ag@ Ag_2_MoO_4_–AgBr composite. *Journal of Hazardous Materials*.

[13] Da Silva M. O., Aquino S. (2018). Resistência aos antimicrobianos: uma revisão dos desafios na busca por novas alternativas de tratamento. *Revista de Epidemiologia e Controle de Infecção*.

[14] Moura J., Freitas T., Cruz R. (2019). Antibacterial properties and modulation analysis of antibiotic activity of NaCe (MoO4) 2 microcrystals. *Microbial Pathogenesis*.

[15] Moura J., Freitas T., Cruz R. (2017). *β*-Ag2MoO4 microcrystals: characterization, antibacterial properties and modulation analysis of antibiotic activity. *Biomedicine & Pharmacotherapy*.

[16] Oliveira C. A., Volanti D. P., Nogueira A. E., Zamperini C. A., Vergani C. E., Longo E. (2017). Well-designed *β*-Ag_2_MoO_4_ crystals with photocatalytic and antibacterial activity. *Materials & Design*.

[17] Chen X., Liu F., Yan X. (2015). Ag_2_Mo_3_O_10_ nanorods decorated with Ag_2_S nanoparticles: visible‐light photocatalytic activity, photostability, and charge transfer. *Chemistry—A European Journal*.

[18] NCCLS (2003). *Methods for Dilution Antimicrobial Susceptibility Tests for Bacteria that Grow Aerobically*.

[19] Coutinho H. D., Costa J. G., Lima E. O., Falcão-Silva V. S., Siqueira-Júnior J. P. (2008). Enhancement of the antibiotic activity against a multiresistant *Escherichia coli* by mentha arvensis L. and chlorpromazine. *Chemotherapy*.

[20] Javadpour M. M., Juban M. M., Lo W. S. (1996). A new method for determine the minimum inhibitory concentration of essential oils. *Journal of Applied Microbiology*.

[21] Salvat A., Antonnacci L., Fortunato R. H., Suárez E. Y., Godoy H. (2001). Screening of some plants from northern argentina for their antimicrobial activity. *Letters in Applied Microbiology*.

[22] Murphy A. B., Murphy A. (2007). Band-gap determination from diffuse reflectance measurements of semiconductor films, and application to photoelectrochemical water-splitting. *Solar Energy Materials and Solar Cells*.

[23] Foggi C. C., Fabbro M. T., Santos L. P. (2017). Synthesis and evaluation of *α*-Ag_2_WO_4_ as novel antifungal agent. *Chemical Physics Letters*.

[24] Noronha V. T., Paula A. J., Duran G. (2017). Silver nanoparticles in dentistry. *Dental Materials*.

[25] Berni Neto E., Ribeiro C., Zucolotto V. (2008). *Síntese de nanopartículas de prata para aplicação na sanitização de embalagens*.

[26] Ali T., Ahmed A., Alam U., Uddin I., Tripathi P., Muneer M. (2018). Enhanced photocatalytic and antibacterial activities of Ag-doped TiO_2_ nanoparticles under visible light. *Materials Chemistry and Physics*.

[27] Chaturvedi S., Dave P. N. (2018). *Nanomaterials: Environmental, Human Health Risk, Handbook of Nanomaterials for Industrial Applications, Micro and Nano Technologies*.

[28] André R. S., Zamperini C. A., Mima E. G. (2015). Antimicrobial activity of TiO_2_: Ag nanocrystalline heterostructures: experimental and theoretical insights. *Chemical Physics*.

[29] Bing W., Chen Z., Sun H. (2015). Visible-light-driven enhanced antibacterial and biofilm elimination activity of graphitic carbon nitride by embedded Ag nanoparticles. *Nano Research*.

[30] Cheng H., Xiong W., Fang Z. (2016). Strontium (Sr) and silver (Ag) loaded nanotubular structures with combined osteoinductive and antimicrobial activities. *Acta Biomaterialia*.

[31] Smekalova M., Aragon V., Panacek A., Prucek R., Zboril R., Kvitek L. (2016). Enhanced antibacterial effect of antibiotics in combination with silver nanoparticles against animal pathogens. *Veterinary Journal*.

[32] Ragàs X., He X., Agut M. (2013). Singlet oxygen in antimicrobial photodynamic therapy: photosensitizer-dependent production and decay in *E. coli*. *Molecules*.

[33] Melo W. C. M. A., Perussi J. R. (2012). Comparando inativação fotodinâmica e antimicrobianos. *Revista de Ciências Farmacêuticas Básica e Aplicada*.

[34] Hakouk K., Deniard P., Lajaunie L. (2013). Novel soft-chemistry route of Ag_2_Mo_3_O_10_ 2H_2_O nanowires and in situ photogeneration of a Ag@ Ag_2_Mo_3_O_10_ 2H_2_O plasmonic heterostructure. *Inorganic Chemistry*.

[35] Liu J., Liu Z., Zhang J., Ma Z. (2020). AgI/Ag_2_Mo_3_O_10_ 1.8 H_2_O: a new photocatalyst working under visible light. *Materials Chemistry and Physics*.

[36] Ribeiro V. A. d. S., Ferrari A. M., Tavares C. R. G. (2020). Fotocatálise aplicada ao tratamento de efluentes de lavanderia de jeans: comparação entre TiO_2_ e ZnO na eficiência de remoção de cor/Photocatalysis applied tolaundry wastewater treatment: comparison between TiO2 and ZnO on the efficiency of color removal. *Brazilian Journal of Business*.

[37] Baneshi M. M., Jahanbin S., Mousavizadeh A., Sadat S. A., Rayegan-Shirazi A., Biglari H. (2018). Gentamicin removal by photocatalytic process from aqueous solution. *Polish Journal of Environmental Studies*.

[38] Chen Q., Liu H., Xin Y., Cheng X. (2013). TiO_2_ nanobelts—effect of calcination temperature on optical, photoelectrochemical and photocatalytic properties. *Electrochimica Acta*.

[39] Serna-Galvis E. A., Ferraro F., Silva-Agredo J., Torres-Palma R. A. (2017). Degradation of highly consumed fluoroquinolones, penicillins and cephalosporins in distilled water and simulated hospital wastewater by UV254 and UV254/persulfate processes. *Water Research*.

